# Improving the Use of Blockchain Technology in Stroke Care Information Management Systems

**DOI:** 10.1155/2022/2642841

**Published:** 2022-09-26

**Authors:** Yuying Yang, Aixia Song, Qing Chang, Hongmei Zhao, Weidan Kong, Qian Xue, Qianlong Xue

**Affiliations:** ^1^Stroke Office, The First Affiliated Hospital of Hebei North University, Zhangjiakou, Hebei 075000, China; ^2^Department of Neurology, The First Affiliated Hospital of Hebei North University, Zhangjiakou, Hebei 075000, China; ^3^Emergency Department, The First Affiliated Hospital of Hebei North University, Zhangjiakou, Hebei 075000, China

## Abstract

Blockchain is a new and popular technology in the digital age. Blockchain technology is referred to as decentralised and distributed digital ledgers, which are called blocks. These blocks are linked together with the cryptographic hashes and are used to record transactions between many computers. No single block can be altered without altering the related blocks. Modification of individual block data is impossible because each block contains information from the previous block. This is the unique strength of blockchain. Timestamps and hashes are some of the important terms when blockchains are considered. Data security is guaranteed with this advanced technology. Blockchain technology finds its application in the healthcare industry with many advantages in a queue. Medical data can be transferred safely and securely for fool-proof management of the medicine supply chain, which helps in healthcare research. Blockchains are used to securely encrypt a patient's information in the event of an outbreak of a pandemic disease. A stroke is referred to as a brain attack, also called cerebral infarction. A cerebral infarction is a sudden stoppage of blood flow in the blood vessels connected to the brain. This study focused on evaluating the application of blockchain technology in Stroke Nursing Information Management Systems. This emerging technology is already in use in the healthcare industry. The patient's data is kept decentralized, transparent, and mainly incorruptible, thus keeping it secured and sharing of data is quick.

## 1. Introduction

Validation and storage are performed using the blockchain data structure. Consensus methods and distributed nodes are typically used together to generate and update data. Both data transit and access are protected by encryption. Smart contracts, which are automated script codes, are being used to build and modify the blockchain [1]. It fosters trust in an untrustworthy competitive atmosphere while costing very little, and blockchain technology is seen as a breakthrough development in computing. As a result of the rapid advancement of new technology, industries all around the world have been reorganised [2]. The blockchain, which is increasingly being used by other firms, is built on encrypted digital currency. It is becoming increasingly clear that blockchain technology has the potential to revolutionise several industries, including medicine and healthcare. Because of blockchain technology, people could witness a major shift in how medical records are processed. Among the many benefits of storing data in a decentralised manner are increased trust, information security, and individual privacy [3]. When it comes to this new technology, there are so many ways in which it may be applied.

One of the hottest blockchain study areas right now is electronic medical data processing. A blockchain can be used to store electronic medical records. If all medical data were kept on the blockchain, it would place a greater load on the network's compute and storage resources [4]. These concerns can be avoided by using a hybrid storage architecture that keeps medical data in a database, and only the index of that data on a distributed ledger like blockchain, which can then be used to locate the data. To help diagnose e-health systems, they came up with the notion of using two different types of distributed ledgers: a private and a consortium blockchain [5]. Custom data structures and consensus methods are required for both types of blockchain. The Electronic Health Record (EHR) sharing protocol was built on two types of blockchains: a private blockchain to store EHRs and a consortium blockchain to store safe indices of EHRs [6]. The privacy and security of patients' medical records must be safeguarded if blockchain technology is to be used. Authorized users can securely exchange data thanks to the blockchain's encryption capabilities. They established a blockchain-based system that enables patients, healthcare professionals, and third parties to securely, interoperatively, and quickly access medical data [7]. The use of smart contracts and cutting-edge encryption methods on an Ethereum-based blockchain has improved data security [8].

Because there is no trusted central authority on the blockchain network, consensus is extremely difficult to achieve. [9]. Prior to encrypting the material, the researchers were able to verify Proof of Word and interoperability for blockchain-based data discovery and access [10]. According to the researchers, the PBFT algorithm was used to construct a blockchain-based solution for patient-to-researcher transfers that maintains privacy [11]. As long as a distributed consensus is in place, medical data can be transmitted safely. A smart contract could be created by utilising the framework. Using hospitals and clinics as miners and verifiers, the Proof of Authenticity consensus method is used [12]. The Hyper Ledger Fabric open-source project uses an open-source framework to implement a permissioned blockchain and provides scalable applications, such as identity verification, peer-to-peer protocol, access control, consensus algorithm, and smart contracts, to support blockchain use cases in electronic medical records sharing [13]. Hyperledger Fabric-based Blockchains can be utilised to govern the use of a mobile health application [14].

There are a few studies on this topic, but blockchain technology has sparked the interest of researchers interested in managing electronic medical data [15]. Despite the importance of technical inquiry into the difficulties of blockchain technology, nothing has been said about the concept, connotation, and management approaches for the expansion of electronic medical records in the contemporary technological environment. For blockchain solutions, the present literature lacks an integrated research framework that focuses on a specific technological difficulty, such as protecting privacy in electronic medical records or improving consensus algorithms [16]. For the most part, blockchain systems are built only on the basis of computer simulations, with no thought given to how they would be used in the real world. According to the findings of the researchers, while considering legal and regulatory limits, very little thought was given to how the answer might be applied in real industrial settings [17, 18]. Although there are numerous ways in which blockchain technology might improve the integrity and efficiency of electronic medical records, the technology itself is not the most significant component of the process.

According to the findings provided here, ERMR data may be shared securely across a distributed network using blockchain technology [19]. This is the first study of its kind. The study's blockchain-based medical data sharing system also has two other features: system controllability and data security levels. With blockchain technology, ERMR administration may be made easier and more cost-effective by addressing the question of how ERMR can be safely shared and gathered while addressing practical issues. There has been a positive impact on healthcare technology and efficiency because of the conclusions of this study [20]. Additionally, this article uses advanced computer technology to provide an industry reference path and to design and develop a path that would help lead to specific blockchain applications in the healthcare and medical industries. Blockchain is more than simply a piece of information technology; it is a unique blend of existing data storage and transmission technologies, like decentralised databases and point-to-point links, with novel algorithms for consensus and encryption [21]. As an alternative to traditional methods of distributing ERMRs, it offers the advantages of open source and programmability, as well as distributed storage and partial decentralisation [22]. Using a peer-to-peer network architecture, the nodes of the blockchain network are connected together. Since the distributed storage system does not have a central node, each of the distributed storage nodes has a copy of all the data [23]. Since all nodes in the system have access to the block data, the blockchain is a distributed and decentralised database. In the blockchain, a data structure organises and stores data. Two new blocks are created when a block's header and body are separated. The block timestamp and difficulty are two pieces of information included in the block header that are necessary when constructing a Merkle tree. A Merkle tree structure is used to store the block's data transactions. Perform hash operations in pairs on all of the leaf nodes to get to the Merkle tree's root [24]. The hash algorithm is a key component of the blockchain. Block transaction data can be obscured by generating a series of hash values with a defined length using the hash function, which is a general term for various different hashing methods (akin to garbled codes). Many algorithms, such as SHA-256, can convert any transaction data string into a 64-character string. People will never be able to figure out what the initial hashing algorithm was [25]. This means that it can be used to protect both personal information and sensitive data by encrypting them, so it can do this. Multifactor Authentication (MFA) including Elliptical Curve Cryptography is compared to the standard technique of conducting online transactions in the suggested framework (ECC). The performance evaluation demonstrates that the proposed framework is both secure and efficient, requiring less time and money to execute encryption and decryption. The reduced computational time is evaluated with a sample dataset to validate the suggested work [26].

## 2. Materials and Methods

In Stroke Nursing, the management of medical information is an important task represented in Figure 1. Safety and security are considered to be important points to be taken care of. The medical data of the patient like treatment taken, medical reports like Electronic Medical Record (EMR), Personal Health Reports (PHR), Electronic Health Report (EHR) are fed into the management cloud. These information are formed into blocks in the blockchain phase. The hospitals are well equipped with wireless sensor networks (WSN). The wireless networking technology helps in sharing the data to the cloud. Light-weighted Deep Learning Models are deployed in transferring the written and typed medical information to the blockchain. The Natural Language Processing (NLP) algorithm is used along with Deep Learning Models for this purpose.

The patient's data are securely encrypted with the help of blockchain. The blockchain data can be accessed from the cloud by the users (patients, doctors, healthcare staff, nurses). Blockchain technology provides an improved way of sharing medical data in a secured manner. The digital health records are securely stored and accessed by authorized users. The identity of the patient is protected in this case. The administration process is well automated by establishing secured contracts between the patients and hospitals with the help of blockchain. The safe arrival of drug shipment and prevention of counterfeit medicines. The blockchains monitor diseases and reports in the case of an outbreak of a pandemic.

Light-Weighted Deep Learning Models are used to predict stroke in patients. Tests like EEG, ECG, and EMG use the sensor technologies to diagnose the patients in treating stroke. The patient's brain activity is monitored with an electroencephalogram (EEG). It is a test that detects electrical activity of the brain using small electrodes attached to the scalp. Electromyography (EMG) is referred to as a process used to measure the activity of the muscle in response to nervous stimulations. An electrocardiogram (ECG) uses sensors that were taped to the chest, arms and legs. The sensors measure the heartbeat. The signals are depicted in a wave pattern that can be monitored on a computer screen. The data from these sensor technology devices are collected and sent through the WSN network to the cloud. The data in the cloud is analysed and stroke prediction is done with the help of AI. These data are sent to the medical practitioners who in turn act quickly and treat the patient immediately. Thus blockchain technology improves the Stroke Nursing Information Management system.

### 2.1. Proposed Work

A neural system identifies the *g* [*k*, *k* + 1] operation as part of the confidence earned via stroke prediction neural network interpretation. Using the period of time given by *k* and also the framework conditions *k* + 1, this should provide *g*(*k* + 1). A stochastic modification module not only increases the authority of the stroke prediction neural network function and *g* is the anticipated possibility of judgments with *g*(*k*) but it also provides a finished result. These definitions are given as.

(1) $$\begin{array}{c} m^{\prime }\left(k\right)=\overset{d}{\underset{k+1}{\sum }}d\left(m\left(k\right)+\overset{k}{\underset{g=1}{\sum }}g\left[k,k+1\right]\right). \end{array}$$

The stroke prediction neural network rule unit *n*_*i*_ is organized for evaluate the stroke prediction neural network guideline. The data *m*(*k*) device is a standard predecessor that receives a unit. Unit  *g* = 1 communicates with the behaviour control. The process is completed with a neutralized combination.

Signs and weightlifting are actual values with input nodes. These indicators are unaffected by the data. The result is substantially equal to the data. The signal *n*_*i*_ may collaborate with truck full to *s*_*i*_ to create such objects as.

(2) $$\begin{array}{c} g=\sum s_{i}n_{i}+\overset{k}{\underset{g=1}{\sum }}g\left[k,k+1\right]\;i=1,2. \end{array}$$

In order to implement the data, necessary data input FL is gathered as.

(3) $$\begin{array}{c} \text{FL}=\overset{s}{\underset{g⟶n}{\sum }}g_{1}+g_{2}=\overset{s=1}{\underset{k=1}{\sum }}s_{1}k_{1}+s_{2}k_{2}. \end{array}$$

The neuron uses its transfer work *f*(*y*)  to calculate the FL is neural network production, which could be a sigmoid function result *f*(*y*) = (1 + *e*^−*y*^)^−1^ is calculated as.

(4) $$\begin{array}{c} f\left(y\right)=\sum f\left(\text{FL}\right)=\int f\left(s_{1}k_{1}+s_{2}k_{2}\right)+\overset{s}{\underset{g⟶n}{\sum }}g_{1}+g_{2}. \end{array}$$

An ordinary deep network is a simple neural net that makes use of redundancy, inclusion, and the sigmoid function *f*(FL).

A set of stroke prediction neural networks was defined for the decision support system employed during DL-based digital stroke nursing information management and system records. These are based on both factual data and stroke prediction neural network information. The following are some neural network examples.

Because, when *G* = 1 completing activities, this mode command technology not only uses the point of entry and the available spectrum and data transfer but it also transmits *h*_(*i*)_ web access.

(5) $$\begin{array}{c} s_{i}^{g}=\overset{Y}{\underset{G=1}{\sum }}\alpha_{i}R\log\left(1+\frac{{\left|g_{i,n}\right|}^{2}Y_{i,n}g^{-n}}{\sigma^{2}}\right)+\sum f\left(\text{FL}\right). \end{array}$$

In the Equation (5), *i* denotes its percentage of internet connectivity bandwidth inhabited by terminal update specific assignments,  *g*_*i*,*n*_ denotes the connection downturn transformation function between access point and terminal; and *Y*_*i*,*n*_ denotes terminal products, *g*^−*n*^ denotes node facility distance, *b* denotes news team loss, and *σ*^2^ denotes interaction noise level. Similarly, the efficiency of *g*_*i*_ downlink data transfer is defined as.

(6) $$\begin{array}{c} d_{i}^{k}=\overset{X}{\underset{g=1}{\sum }}\beta_{i}B\log\left(1+\frac{{\left|g_{n,i}\right|}^{2}X_{n}g^{-b}}{\sigma^{2}}\right)+\overset{s}{\underset{i=1}{\sum }}s_{i}^{g}+\overset{n}{\underset{i=1}{\sum }}{\left|g_{n,i}\right|}^{2}X_{n}g^{-b}, \end{array}$$

which, the  *β*_*i*_ represents the proportion of the throughput frequency range occupied by a terminal capable of receiving tasks,  *g*_*n*,*i*_ represents the link economic downturn correlation between entry point and terminal, and  *X*_*n*_ represents the foundation network's connection speed.

The fundamental goal of optimizing an online healthcare system based on edge devices is to achieve the task information technology offload framework with the shortest time delay, which is constituted of two bits: digital technology time delay solely on local and frame clients.

If task  *n*_*i*_ also is not offloaded to a network edge, it is approximated on the gateway as well. The time difference between doing the jobs geographically is denoted as.

(7) $$\begin{array}{c} X_{i}^{n}=\overset{n}{\underset{k=1}{\sum }}\frac{g_{i}}{g_{i}^{k}}+{\left|g_{n,i}\right|}^{2}X_{n}g^{-b}+\overset{n=1}{\underset{i=1}{\sum }}\frac{{\left|g_{n,i}\right|}^{2}X_{n}g^{-b}}{\sigma^{2}}. \end{array}$$

In where *g*_*i*_^*k*^ signifies the terminal  *g*_*i*_ communication processing's ability to organise tasks regionally. As a result, the entire time delay identified by *g*_*i*_ researchers at the local scale is depicted as.

(8) $$\begin{array}{c} g_{i}^{m}=\underset{m\in g}{\sum }\left(1-\alpha_{i}\right)g_{i}^{m}+\overset{n}{\underset{k=1}{\sum }}\frac{g_{i}}{g_{i}^{k}}+{\left|g_{n,i}\right|}^{2}X_{n}g^{-b}. \end{array}$$

Therefore in situation, we connect the approaching information to a neuron using various activities including a *t*-norm or even a *n*_*i*_-conorm; these results are calculated using Equation (9) which can be termed as a hybrid artificial neuron.

(9) $$\begin{array}{c} g_{i}^{n}=\overset{n=1}{\underset{i=1}{\sum }}\frac{m_{i}}{g_{i}^{n}}+\overset{n}{\underset{k=1}{\sum }}\frac{g_{i}}{g_{i}^{k}}+{\left|g_{n,i}\right|}^{2}X_{n}g^{-b}. \end{array}$$

As a result of these modifications, stroke prediction neural network neural planning is dependent on stroke prediction neural network increasing computational. As shown in the graph, the frequency band delay time is proportional to the amount of data obtained and also the network capacity for data transfer function.

(10) $$\begin{array}{c} g_{i}^{n}=\overset{k}{\underset{i=1}{\sum }}\frac{g_{i}}{b_{i}^{k}}+\underset{m\in g}{\sum }\left(1-\alpha_{i}\right)g_{i}^{m}. \end{array}$$

A set of neural networks was described for stroke nursing information management with health system of care employed in deep learning based stroke nursing information management with health system care. These have been backed not only by facts but also by stroke prediction neural network data, and the server's calculation time is comparable to a magnitude of a clear stands and the server's computing capabilities:

(11) $$\begin{array}{c} b_{i}^{f}=\overset{X}{\underset{i=1}{\sum }}\frac{f_{i}}{X_{i}}+\overset{n}{\underset{i=1}{\sum }}\left(1+\frac{{\left|g_{i,n}\right|}^{2}Y_{i,n}g^{-n}}{\sigma^{2}}\right). \end{array}$$

A temperature sensor is a small chip that measures the body's temperature in degrees Celsius. The temperature is displayed in this framework of body temperature controller which is expected to function far better than a linear temperature controller. As a result, the time spent offloading assignment *s*_*i*_ to the edge devices is sent as.

(12) $$\begin{array}{c} s_{i}^{n}=\overset{s=1}{\underset{i=1}{\sum }}s_{i}^{c}+s_{i}^{h}+s_{i}^{f}+\overset{Y}{\underset{G=1}{\sum }}\alpha_{i}R\log\left(1+\frac{{\left|g_{i,n}\right|}^{2}Y_{i,n}g^{-n}}{\sigma^{2}}\right). \end{array}$$

Respiratory arrest, cardiac condition, vagal convulsion, and the pressure gauge are all monitored urgent requirements. As a consequence, the time duration associated with the task of discharging *s*_*i*_ to the edge device is communicated as.

(13) $$\begin{array}{c} X_{i}^{n}=\overset{n=1}{\underset{i=1}{\sum }}\alpha_{i}s_{i}^{n}+\overset{s=1}{\underset{i=1}{\sum }}s_{i}^{c}+s_{i}^{h}+s_{i}^{f}. \end{array}$$

The pulse rate appears to be the most important sign of vital medical behaviour with stroke nursing data management for health-care system fitness. A pulse-rate sensor is the most commonly explored sensor in the field of patient outcomes and management:

(14) $$\begin{array}{c} \min\;g=\overset{n}{\underset{i=1}{\sum }}\left(g_{i}^{n}+d_{i}^{n}\right)+\overset{n=1}{\underset{i=1}{\sum }}X_{i}^{n}. \end{array}$$

It is being used to assess pulse rate including more complex disorders such as a heart attack. The sensor activates whenever an object *f*1 places its finger directly on the information display. The outcome is displayed on the input panel:

(15) $$\begin{array}{c} s.t.f1:\underset{h_{i}\in d}{\sum }m_{i}\leq m_{y}+m\left(k\right)+\overset{k}{\underset{g=1}{\sum }}g\left[k,k+1\right]. \end{array}$$

The deep learning smart stroke nursing information management scheme is necessary for health system care client administration and monitoring. The proposed *f*2 technique (Equation (16)) benefited from a neural network architecture that is simple to use and enforce for decision making.

(16) $$\begin{array}{c} f2:\underset{g_{i}\in d}{\sum }\alpha_{i}\leq 1+\underset{h_{i}\in d}{\sum }m_{i}\leq m_{y}+m\left(k\right). \end{array}$$

The organization of the *f*3, proposed system as in Equation (17), is unusual in that it uses not just sensory data but also a stroke prediction neural network decision-making process.

(17) $$\begin{array}{c} f3:\underset{g_{i}\in d}{\sum }\beta_{i}\leq 1+\underset{h_{i}\in d}{\sum }m_{i}\leq m_{y}+g\left[k,k+1\right]. \end{array}$$

Since the *f*4 in Equation (18) is to reduce an energy economy's delay time, attractiveness is characterised in terms of the time delay, and reduced time latency corresponds to higher athletic.

(18) $$\begin{array}{c} f4:\overset{n=1}{\underset{i=1}{\sum }}m_{i}^{n}\geq 0,\forall i\in d+\overset{d=1}{\underset{i=1}{\sum }}d_{i}=\frac{1}{g_{i}}. \end{array}$$

The Equation (18) is used to compute the *d*_*i*_  strength and endurance value.

## 3. Result and Discussion

Figure 2 depicts the variance in data acquired by the temperature sensor, pulse rate sensor, and blood pressure sensor. The data distances are also calibrated using Table 1 and Table 2. The input data is captured and calibrated before stroke prediction neural network is utilised to make decisions about the patient's status in the second step. Table 1 displays the scaled output values for the user-entered data.

Cardiac arrest, blood clot, vagal convulsion, and the pulse sensor are all monitored emergency situations. The key determinant for critical health issues as well as skin fitness is heart rate. The pulse rate receiver is the most extensively used and research detector in patient monitoring and safety.

Sensors for temperature, pulse rate as well as blood pressure are used in this technique to assess the patient's condition under analysis (Figure 3). The scheme used a body of knowledge and stroke prediction neural network system for decision support for patient care, supervising as well as management to determine possible circumstances and cures. The stroke prediction neural network technique also tried to improve the performance of this system for patient monitoring and treatment in terms of the time, cost, and workforce consumption.

Within a week of receiving information collected using sensors and transferred via smart device, the patient document measure is generated solely on the server. The data is separated into three sections: patient data, geographical information, and the patient's ailments. Table 2 only contains information about the places where we choose to test the model. Testing will be done in approximately eight different locations. The location of the chosen establishments and the testing time frame range.

The technique incorporates patient monitoring to sensors and offers great precision and efficiency benefits over current systems (Figure 4). The investigation was conducted on a small sample population and proven to be efficient, exact, and purposeful. So far, the technique has been generalized, and it is conceivable to tailor it to more serious conditions such as operating room patients, intensive care patients, newborns, and patients with considerably more complex medical histories.

Temperature ranges ranging from 100°F to 105°F have been used to identify four categories of temperature measurements (there is no fever, fever, a fever is prevalent, and exceptionally high fever). It has three pulse rate classes for a typical human being: low, normal, and high. Low pulse rate is defined as less than 60 beats per minute. Normal pulse rate is described as a pulse rate between 60 and 100. A pulse rate more than 100 is considered to be a high pulse rate. The difference in blood pressure from normal to abnormal is depicted in Table 3. A blood pressure reading of 120/80 mmHg is considered normal. High blood pressure is defined as a pulse rate of 129–140/81–89 BP. Extremely high blood pressure.

A first patient results monitoring and control system that uses a stroke prediction neural network method to identify patients' symptoms as well as prospective therapies (Figure 5). The results in Tables 4 show that when sensors and recommender systems were used, this technique performed well. The neural network system's judgment process increases the method system's efficacy and practicality. This system is distinct in that it makes suitable decisions using sensors and a DL-based architecture.

Table 4 illustrates a patient's information gathered on that website after receiving data collected via sensors and transferred via smart device. The report is broken into three sections: patient data, sensor information, and also the patient's ailments.

The choice is made by the neural network system, and indeed the stroke prediction decision accuracy is measured (Figure 6). The accuracy of the suggested service ranges from 97 percent to 100 percent, according to Table 5. It shown that the proposed system follows the rules defined for patient safety along with managed services decision making.

Also to time it took the general practitioner to respond to the inquiries. The proposed technique is a low-cost and efficient option for those living in rural places; it may be used to detect if they have a major health problem and treat them appropriately by contacting neighboring hospitals. Using detectors and decision support tools in healthcare is a novel approach, and Table 5 demonstrates how it decreases time limitations when compared to typical telemedicine methods. Using blockchain technology in the healthcare sector has many advantages, including decreasing wait times. Medical data can be transmitted safely and reliably in healthcare research to guarantee an error-free medication supply chain. Blockchain can be used to securely encrypt patient data in the event of a pandemic disease outbreak. A stroke is a type of brain attack, often known as an infarction. A cerebral infarction is an abrupt stoppage of blood flow in the brain's arteries. The inquiry into the application of blockchain technology in this article focuses on stroke nursing information management systems.

## 4. Conclusions

The digital age has given rise to a new and popular technology is called blockchain. Decentralized digital ledgers, or blocks are used to describe blockchain technology. The cryptographic hashes link these blocks together, allowing them to serve as a record of transactions involving multiple machines. When discussing blockchain, concepts like timestamps and hashes are critical. With this cutting-edge technology, you can rest assured that your data is safe. There are numerous benefits to using blockchain technology in the healthcare industry, such as reducing wait times. In healthcare research, medical data can be sent securely and reliably to ensure a flawless supply chain for medicines. In the case of a pandemic illness breakout, patient data can be encrypted securely using blockchains. A brain assault or infarction is referred to as a stroke. A sudden halt in blood flow in the brain's arteries is known as a cerebral infarction. Stroke nursing information management systems are the focus of this article's investigation into the use of blockchain technology. This study helps in analysing the security aspects of storing patient information in stroke nursing. The results shown that the proposed system follows the rules defined for patient safety along with managed services decision making.

## Figures and Tables

**Figure 1:** Architecture diagram of the proposed system.

**Figure 2:** Performance analysis for sensor data difference is obtained in stroke nursing identification for the blood pressure.

**Figure 3:** Accuracy of results of stroke prediction with neural networks algorithm based decision making.

**Figure 4:** The dependability of the outcomes of neural network-based stroke prediction decisions.

**Figure 5:** Performance analysis for stroke prediction data from sensors will be used in the deep learning experimentations.

**Figure 6:** The outcomes of decision-making based on stroke prediction neural network.

**Table 1:** Result analysis for information on experimental investigation as well as data analysis.

No	Location ID	Stroke nursing information management	Blood pressure selective sample	Stroke testing period
1	Loc-4	19	5	Oct 2021
2	Loc-1	25	3	Nov 2021
3	Loc-7	37	2	Jan-20201
4	Loc-3	48	4	July – 2021
5	Loc-5	33	5	Sep-2021
6	Loc-2	16	3	Aug-2021
7	Loc-6	65	2	Feb – 2021

**Table 2:** Report from the patient information.

Patient data		Sensor information	
Name of the patient	ABC	The body's temperature	99.96°F
CNIC patient	33165674548246	The rate of pulse	87BPM
Address of the patient A	XYZ	High blood pressure	97/140

**Table 3:** Temperature ranges.

Parameters	Temperature ranges	Classes of pulse rate	Classes of blood pressure	Class
Temperature (°F)	<99 99–101 101.1–103 >103.1			There is no fever. Fever A fever is prevalent. Extremely high fever

Pulse rate (NN)		>100 61 to 100 <60		Increased Normal Reduced

BP (HG)			<110/<70 120–110/80–70 120/80 130–139/80–89 >140/>90	Incredibly low Low Ordinary High Extremely high

**Table 4:** Result analysis for stroke prediction data from sensors will be used in the deep learning experimentations.

No	Temperature (°F)	Pulse rate (%)	Blood pressure (BP-low)	Blood pressure (BP-high)
1	104	61-100	87	180
2	100	70	100	145
3	104	110	95	127
4	103	106	89	143
5	95	107	82	132

**Table 5:** Stroke prediction sensor data measurement using a neural network technique.

No	Temperature	Pulse rate	Blood pressure	Neural network decision	Accuracy (%)	Percent error (%)
1	Normal	High	Low	High	99.43	4.6
2	High	Normal	High	Medium	94.32	6.6
3	Normal	High	Medium	Low	88.64	6.5
4	Low	Low	Low	Low	95.88	14.64
5	High	High	High	High	96.42	12.99
6	Normal	Medium	Medium	High	98.98	8.4
7	Medium	Low	Low	Medium	94.66	9.5
8	Very high	High	High	Low	93.97	8.65
9	Medium	High	Low	High	88.65	9.65
10	Very high	Medium	Low	Low	87.98	9.35

## Data Availability

The data used to support the findings of this study are available from the corresponding author upon request.
